The article "IoT-Based Wearable Devices for Patients Suffering from Alzheimer Disease" was published in 2022. Journal: Contrast Media Mol Imaging.

# IoT-Based Wearable Devices for Patients Suffering from Alzheimer Disease

**DOI:** 10.1155/2022/3224939

**Published:** 2022-04-22

**Authors:** Waleed Salehi, Gaurav Gupta, Surbhi Bhatia, Deepika Koundal, Arwa Mashat, Assaye Belay

**Affiliations:** ^1^Yogananda School of Artificial Intelligence Computer and Data Sciences, Shoolini University, Bajhol Solan 173229, HP, India; ^2^Department of Information Systems, College of Computer Science and Information Technology, King Faisal University, Al Hasa, Saudi Arabia; ^3^Department of Systemics, School of Computer Science, University of Petroleum & Energy Studies, Dehradun, Uttrakhand, India; ^4^Faculty of Computing and Information Technology, King Abdulaziz University, Rabigh, Saudi Arabia; ^5^Department of Statistics, Mizan-Tepi University, Ethiopia

## Abstract

The disorder of Alzheimer's (AD) is defined as a gradual deterioration of cognitive functions, such as the failure of spatial cognition and short-term memory. Besides difficulties in memory, a person with this disease encounters visual processing difficulties and even awareness and identifying of their beloved ones. Nowadays, recent technologies made this possible to connect everything that exists around us on Earth through the Internet, this is what the Internet of Things (IoT) made possible which can capture and save a massive amount of data that are considered very important and useful information which then can be valuable in training of the various state-of-the-art machine and deep learning algorithms. Assistive mobile health applications and IoT-based wearable devices are helping and supporting the ongoing health screening of a patient with AD. In the early stages of AD, the wearable devices and IoT approach aim to keep AD patients mentally active in all of life's daily activities, independent from their caregivers or any family member of the patient. These technological solutions have great potential in improving the quality of life of an AD patient as this helps to reduce pressure on healthcare and to minimize the operational cost. The purpose of this study is to explore the State-of-the-Art wearable technologies for people with AD. Significance, challenges, and limitations that arise and what will be the future of these technological solutions and their acceptance. Therefore, this study also provides the challenges and gaps in the current literature review and future directions for other researchers working in the area of developing wearable devices.

## 1. Introduction

The growing prevalence of dementia presents a major challenge to global health at different levels. Hurd and colleagues (2013) estimated at the financial level that dementia and, specifically, AD are among the diseases that are most expensive for the western region with a $160 billion per year price tag [1, 2]. Alzheimer's is a kind of disease that typically and slowly progresses in three main stages such as early, middle, and moderate or late [3]. Since this disease is affecting people in several different ways, so in that case, every affected person may experience different symptoms or go through the stages differently [3], as in Table 1 a short description of the activities that can be affected by AD is given.

The article "IoT-Based Wearable Devices for Patients Suffering from Alzheimer Disease" was published in 2022. Journal: Contrast Media Mol Imaging.

A rapid digital revolution is taking place in the twenty-first century [4]. The Internet of Things is a buzz term in recent years very commonly called IoT. It is a relatively new idea that allows real-world physical devices or entities to be managed remotely via the Internet. We are witnessing the IoT applications it is used and how it serves humans in many aspects of life; nowadays, the applications such as remote controlling of smart homes, natural disasters alerting, health monitoring of patients, and location tracking. [5]. IoT generally refers to anything that can communicate and exchange data with other devices across a network infrastructure. Here the objects or things can be any embedded systems or sensors that connect with other systems to capture data such as the heart rate of a patient, location information, image recognition, and movements.

The wearable device is one of the major driving technologies of the IoT. Similarly, in entertainment, industrial logistics, sports, and many other fields, wearable computing has implemented and introduced new techniques, more productive processes, and creative goods [6]. However, no other sector, with interests ranging from well-being and prevention of disease to chronic patient care and various other disciplines in medical, anticipates and incorporates wearable technology as widely as healthcare [7] since a wearable IoT gadget combined with a mobile application could be a viable solution for healthcare services, acting as a patient's intelligent personal assistant.

Wearable assistive technology is the term that is used to define systems or devices that enable individuals with physical or communication and cognitive disabilities to improve the quality and capabilities of their life. The advent of wearable technology in recent years has motivated and allowed professionals in the healthcare sector to look beyond the clinic or office to help in identifying and detecting health risks, tracking or monitoring the development of diseases, for instance, patient with Alzheimer Disease (AD), and offer therapy or guidance [7].

The use of wearable devices has been adopted by many people, but we still need to involve IoT with more advanced AI-based techniques [8] for improving the quality of people with Alzheimer's [9].

The article "IoT-Based Wearable Devices for Patients Suffering from Alzheimer Disease" was published in 2022. Journal: Contrast Media Mol Imaging.

In this study, we focus on wearable devices used specifically by AD patients that can also at the same time help their caregivers. The reason this study focuses on wearable devices is that rising healthcare expenses are a major concern; as we defined in the above section, wearable devices are sensors that can be used for remotely collecting health-related data. An example, a sensor passively collecting data on a person's physical activity is an accelerometer incorporated in the form of a wristband [10]. These devices are designed to monitor continually and convey data in real-time or on an ad hoc basis, and they have the potential to become an important component of the future of healthcare research development.

Medical imagings such as Positron Emission Tomography (PET), Magnetic Resonance Imaging (MRI) and so forth have shown a promising earlier detection and prediction of the disease. Currently, due to invasive nature and the cost of these tests, they are limited to research applications [11]. These constraints make it impossible to test an individual repeatedly and frequently, especially in the early stages of presymptomatic disease [12]. IoT-based sensors and wearable technologies have the potential to overcome these constraints, and their use in AD diagnosis has piqued attention [13]. These technologies provide unique services in an economical fashion due to the following reasons [11]:

- Use of such technology by a large number of people
- Development and the variety of onboard sensors
- This is the nature of such type of sensors, which are specially designed to investigate physical and cognitive symptoms
- Although these gadgets are increasingly used by wide sectors of the population, this can have a major impact in healthcare system load, and to extremely lower the burden to the caregiver of a patient.

This study provides a concise study of IoT-based devices such as wearable assistive devices for AD patients and the simple approach to wearable device applications in healthcare for improving the quality of life of AD patients and to evaluate the previous research effort to demonstrate the potential use of these technological solutions for people suffering from the disease. Another main purpose of the study is to provide information on how these wearable devices can be used, what are the different functionalities they can offer, how can they help the patient and their caregivers. A wide range of advantages of using IoT-based sensors under various approaches is discussed. Furthermore, it is required to be pointed out that the use of these devices, however, shown challenges about durability, acceptability, ease of use. The following research questions are used as guidelines a guideline:

- What drives the adoption of wearable devices?
- How effective are the applications of IoT-based wearable devices in patients with Alzheimer's disease?
- Can these technological solutions ease the burden of caregivers of AD patients in the future?
- Do these technological solutions with the use of some algorithms such as machine and deep learning help in more detection and monitoring of AD?

The article "IoT-Based Wearable Devices for Patients Suffering from Alzheimer Disease" was published in 2022. Journal: Contrast Media Mol Imaging.

The organization of this study is as follows: an introduction and the research questions guidelines are given in the first section. The second section described the IoT and wearable devices concisely. Afterward, the literature review is done on various recent works in the field of IoT-based wearable devices for AD patients. Lastly, the result and discussion are done and followed by the conclusion section, and future scopes are suggested.

## 2. Materials and Methods

For achieving the research objectives, a review approach was used on the articles that are published in the area of wearables and IoT technologies and their applicability in elderly Alzheimer's patients. The study and process of targeting the papers are illustrated in Figure 1. Three large digital databases were chosen and searched to improve the odds of getting the best search results. In accordance with previous research studies [14, 15], researchers should always avoid scanning a single database for the literature in a review study; not a single database is likely to include all relevant papers; hence, supplemental searches are required [16].

### 2.1. Criteria for Inclusion

- Papers are published through a conference or a journal, and the text is written in the English language
- The primary aim comes in various technological solutions in healthcare, such as devices, applications, algorithms, and methods
- The technological solutions that are IoT-based and focused for Alzheimer's patients are considered

The case-control of these studies covers diagnosis, monitoring, adherence of medication, and tracking of AD patients. A flowchart is constructed for the identification of articles as follows in Figure 1.

In Figure 1, during the research and obtaining of papers, we have come across 95 papers that are collected from the various scientific sources. After that, we categorized papers in two groups important and not important based on each paper's abstract and conclusion sections, and the irrelevant and duplicate records of 71 have not been considered further. On the remaining research papers, a full-text reading of the paper is done, and 14 papers are excluded in this stage; finally a total number of 10 research-relevant articles are put together for further study.

The article "IoT-Based Wearable Devices for Patients Suffering from Alzheimer Disease" was published in 2022. Journal: Contrast Media Mol Imaging.

## 3. Literature Review

Identifying and meeting the needs of people with cognitive disabilities is crucial for anyone, but it is particularly necessary for those who live alone, with the increased number of aged population around the world [17], the less support and stand from the family members, and a higher cost of formal look after of the patient. Such needs can be addressed by IoT-based wearable systems and enabling technologies and have the potential to do better far beyond them.  Figure 2 gives a view of how these devices have emerged over the past years.

In recent years, various IoT-based and wearable assistive devices are developed and carried out for patients with AD. These devices are implemented and designed in different forms such as locating systems, tracking, and monitoring of the patients. The main aim behind all this is to ease the burden of the caregivers and help the patients and provide a convenient life for them. Ahmed and Al-Neami et al. [19] designed and developed an electronic device known as a smart biomedical assistant in which the aim is to provide continual monitoring of the AD patient's stability state that has the capabilities of reminding the patient automatically of the time of medication, showing the location on the map, and another very important feature that is a button that calls for an emergency case. The device is designed in such a way that one is wearable for the patient and the other one is used by the caregiver that is an IoT platform application that allows communication between the patient and the caregiver. The wearable device contains a global positioning sensor (GPS), motion unit sensor, sensor, and microcontrollers for heart rate and a display of LCD. Roopaei et al. [20] developed IoT-based wearable assistive glasses, and a deep learning approach is used and embedded for the AD patients. This ambient intelligence is based on facial perception for patients with memory difficulties. These face reminder glasses try to assist the patient in recognizing and identifying the people in a patient's family, colleagues', friends, and attempt to help the patient and improve their social skills via a visual understanding of various facial images of the patient's friends, family, and colleagues. For extracting the features of various facial images, the deep learning model is used, and an embedded personalized database is used for matching the facial images. Approximately 90.68% accuracy is achieved by the framework on a labeled face in the Wild dataset for verification of the faces. In another study, Takpoe et al. [21] presented a cost-effective solution of an intelligent assistive health system that can help elderly AD patients in medication adherence. They developed this intelligent assistive health system to give an audiovisual alert to the patients with memory loss disability to achieve medication adherence so that the users can take their right medication doses at the right time through the Liquid Crystal Display (LCD) being used in the system. Furthermore, the physician keyed in the prescriptions of drugs, and nonvolatile memory is used in the system to store the medication schedule. They also used a Subscriber Identity Module (SIM) and an integrated GSM modem so that the system can automatically send an alert message to the physician through an SMS in any case of nonadherences. Similar to the above-proposed system in this study, Oliveira et al. [22] developed an environment aware system in which this device is a wearable waist belt that is used for monitoring the environmental humidity and temperature, the location of the patient using GPS, and the movements of the patients as well. The devices are designed in such a way to send the information to the server and also to the caregiver through an SMS so that the caregiver can get access using an android application which is developed for the smartphone. Thus, the system serves as surveillance over the patient's status. Another monitoring device is designed and developed by Cazangiu et al. [23] for patients suffering from Alzheimer's to monitor their health parameters. A single sensor is used for environmental temperature, hearth pulse, and atmospheric pressure, it also generates an output in a screen to display all those health parameters that are used in the system. Furthermore, using a Bluetooth connection, the parameters can be displayed in a smartphone. Zellefrow et al. [24] presented a wearable solution that monitors and tracks the AD patient known as Halcyon along with a connected assistive indoor platform, which aids AD patients during the daily routine. The system contains four basic components: instruction assignments, detection of patient's engagement with any home appliances, instruction delivery, and tracking of the patient movement, and also, the system generates the patient's activities to the caregiver as a timed log. This system is customizable and prerecorded with the instruction given by the respective caregiver on how to do the routine activities. In this study, the authors Omar et al. [25] designed and developed an integrated autonomous system that includes all the necessary features, unlike the previews papers the features are included such as a reminder for medicine taking, monitoring the heart condition, constantly monitoring of the patient, and finding lost patient's items. In a single system, all the features are integrated, and second, to utilize those features efficiently, a mobile application was also developed. Hegde et al. [26] proposed and developed an autonomous, embedded low-cost wearable device using a concept called geofencing and GPS for tracking the real-time location that can help a caretaker in tracking the AD patient. The system then sends a text message real-time update to the caregiver or family member's mobile number. The alert is sent to the caregiver or a family member when the patient moves out of a safe area and following to that an update of such a situation even is sent after every 5 minutes. Gacem et al. [27] developed a pair of smart glasses that is equipped with a screen of Augmented Reality (AR) that is utilized in this study for performing the basic functions of a caretaker or caregiver and provide the features to the patients which can reduce the caregiving costs and increase the independence of the patient. The main features are the location and detection of misplaced objects and to help out the patient's location where they have been seen last, identifying and showing the relatives and friends names on the AR screen, monitoring the patient all the time if the patient lost his or her way, and the AR screen displays the way home and at the same time, the caregiver receives the location of the patient by an SMS, also in case the patient removes the glasses, detecting and predicting the cause of removal, and giving notification to the caregiver the patient's location and its predicted cause. Chen et al. [28] similar to above cited work in this study also utilized smart glasses; they have proposed a warning system for behavioral difference for dementia warning and early depression. The system is made of three parts smart glasses, cloud-based platform, and an indoor trilateration position that is BLE-based. This wearable device can be useful in recognizing daily movements such as running, walking, standing, lying down, sitting, and many other movements, and these parameters are obtained by a microelectromechanical system sensor (MEMS).

The article "IoT-Based Wearable Devices for Patients Suffering from Alzheimer Disease" was published in 2022. Journal: Contrast Media Mol Imaging.

As we reviewed much-related research work, we have seen that none of them have developed a final wearable product to the market as shown in Table 2 Since some of the paper proposed models, some have developed prototypes to test the proposed work.

Sensors are one of the major and significant components of the IoT-based devices and wearables, and there are many sensors available in the market that are designed for the different specific purposes as detailed in Table 3 that depict what are the different types of sensors used in reviewed wearable devices.

The form factor is one of the main parts when it comes to wearables; as these devices are to be worn by AD patients considerable attention is required to build the wearable devices that will be acceptable and user friendly to the users. As shown in Table 4 we can observe that much work has been done, but when it comes to their design aspects, they are all facing the similar issues in which many of them test the prototype and get not so good feedback about the size, shape, design, and so on.

Table 5 shows various wearable devices with respect to the use of location tracking technology.

Table 6 shows different services and features provided by each wearable device.

When we talk about IoT that is where another important thing come to exist, that is the connectivity of various devices, how they communicate, send, and receive data, and most importantly, are these wearables integrated with some kinds of mobile application, Web-based application, Cloud, etc., in which these are the things that give more features so the patient and, most importantly, their caregivers and the doctor can benefit from them in assisting the patients. The user interface of each device is compared in Table 7.

Table 8 gives an overview of the contrast between various studied wearable devices, with respect to their availability, cost, sensor, IoT, connection, and their form factor. And in Table 9 a complete comparison has been made based on the various features with respect to each device.

Based on various features of each wearable device, a comparison chart is made in Figure 3.

## 4. Basics and Background: IoT Applications in Healthcare Industry

To begin with this new era of technology which is the IoT, first we need to understand the basic backbone of this technology that is Wireless Sensor Networks (WSN). The different aspects of IoT-based devices in digital health are described in Figure 4.

### 4.1. Wireless Sensor Network

Wireless Sensor Networks (WSNs) have emerged as a result of recent advancements and developments in wireless networks and electronics. WSNs have been hailed as one of the most transformative technologies in recent years that can change the future. WSN is a type of network that consists of interconnected devices, which are commonly known as nodes used to wirelessly communicate with each other to collect data of their environment [29]. Small and low battery-powered with minimal computing and radio communication capabilities make up these networks. This technology has been rapidly developing and plays an important role in different domains such as environmental, industrial operations, infrastructures, and healthcare.

The article "IoT-Based Wearable Devices for Patients Suffering from Alzheimer Disease" was published in 2022. Journal: Contrast Media Mol Imaging.

WSN advancements have opened new possibilities in healthcare systems. Medical gadgets have been infiltrated by sensor-based technology, which has replaced hundreds of wired, connected devices in hospitals [30]. As we see the rapid growth of these technologies in recent years, we have witnessed a vast number of wireless devices has been adopted and integrated into the existing medical infrastructures.

### 4.2. Internet-of-Things

IoT refers to a network of linked devices that can use embedded sensors and communication protocols to collect and share data. In general, any kind of device that can connect to the network or Internet is considered to be part of the term called IoT [38]. For example, sensor systems, wearable health monitors, smart home security systems, smart factory equipment, connected appliances.

The difference between the IoT and WSN is all the sensors in an IoT system communicate their data straight to the Internet. A WSN, on the other hand, does not have a direct Internet connection. Rather, the numerous sensors are connected to a router or central node [39]. The data from the router or central node can then be routed as desired. Nowadays, IoT applications can serve in many areas of our lives, for example, alerting in natural disasters, remotely controlling smart homes, tracking of the location [5], and most importantly monitoring health. Even though WSNs and IoT technologies have grown in popularity and acceptance, there are still major risks attached such as limitations in terms of battery life, processing capacity, and bandwidth constraints. More importantly, security, any attacks on control, availability, and privacy can all be targets.  Figure 5 described how digital technologies are used in the society and healthcare sector to enhance and improve the living quality of patients with different kinds of diseases [40, 41], delivering good healthcare services, more personalized and precise medicine, and clinical support.

### 4.3. Wearable Technology

Wearable devices are the next breakthrough in the world of technology, following the advent of smartphones. Wearable devices or wearable technology is a category of electronic devices that can be generally defined as devices that can be used to be worn externally as an embedded or accessory in the person's clothing or implanted in the person's body or even can be tattooed in the skin of the body [42]. These kinds of devices are usually used on a real-time basis to track the information. These devices contain motion sensors that are capable of taking day-to-day movement or activity snapshots and synchronizing that information with other devices such as laptops or mobiles [43], as shown in Table 10 a brief description of the basic components of an intelligent wearable device is given.  Figure 5 depicts the various main components of a typical intelligent wearable system.

The article "IoT-Based Wearable Devices for Patients Suffering from Alzheimer Disease" was published in 2022. Journal: Contrast Media Mol Imaging.

Wearable devices are an example of IoT, which is very useful and have been an integral part of the health and medical industry as shown in Figure 6. For instance, Smart Shirts {Formatting Citation} which are used for monitoring the well-being and health condition of a patient and send the information to the caregiver in a real-time manner. Wearable technologies are comprised of small [44, 45] embedded devices that are used to

1. connect and interact with their environment using a variety of sensors,
2. processing and storing the information, and
3. transferring the data wirelessly to the desired destination for further analysis and processing.

Wearable devices are used to collect data about a person's health, such as

1. Blood pressure
2. Counted steps
3. Burned Calories
4. Time spends in exercise
5. Physical strain [46].

## 5. Challenges and Limitations

Our review from the recent work identified the papers in which they proposed and developed assistive wearable technologies, and we have seen both basic and advanced devices, with their potential applications used for the care of AD patients in different ways and functionalities. Based on the review of literature in Section 3 of this study, the majority of the proposed assistive IoT-based tools focus on reducing the burden for the caregivers and services for individuals or elderly. Some of the developed systems or devices are also designed with detection mechanisms that are experimented with various methodologies of artificial intelligence (AI) such as classification algorithms, deep learning, and machine learning. It is obvious that these new AI-based techniques and algorithms can really impact and increase the capability of IoT-based wearable devices.

Some of the main limitations and advantages of this technological solution for Alzheimer's patients are listed and described below.

Advantages
  - Advancement of social liability.
  - Increased patient's safeness.
  - Disability offsetting of AD patients.
  - Possibly declining treatment costs.
  - Prolong the self-dependency of the patient at the residence.
  - Improved physical and psychological health of the patients.
  - Lastly, possible saving of money on expensive treatments for the community.
Major limitations:

- Deficiencies in the observance of cultural and social differences.
- Lack of evidence on a clinical basis.
- Primary financing is required.
- Concerns regarding the privacy and security of the data.

The article "IoT-Based Wearable Devices for Patients Suffering from Alzheimer Disease" was published in 2022. Journal: Contrast Media Mol Imaging.

There can be a negative reception risk by both caregivers and patient. A complete comparison of all the studied papers is put together in Table 11 with their future scope and limitations.

## 6. Conclusions and Future Trends

Wearable computing is changing the face of digital health in a variety of ways. First and foremost, these wearables are facilitating a shift away from the traditional IT-centralized systems for storage, processing, creation, and management of health-related data into a completely new model era, which is distributed data sharing with patients and the caretaker or the doctor. Second, the integration of wearables and IoT and the data they generate is leading us to use some of the powerful AI techniques for better treatments and automated diagnosis.

A personalized healthcare system is achievable using wearable computing technologies and enables information-sharing through distributed information environment. It also promotes the development of new health information and the development of more effective preventative measures. However, realizing the potential of wearable technologies and digital healthcare would contribute to numerous concurrent technology advancements.

This is an overview of the various technological solutions that are designed and developed for assistive wearable technologies by various researchers for patients suffering from Alzheimer's disease. The aim was to study the recent technological solutions and IoT-based wearable assistive devices accessible in the current time for helping the caregiver and assisting of the AD patients. Based on the current state of potential IoT and wearable applications, it is clear that the future healthcare technologies will rely substantially on the current research.

The limitations of the current research should be addressed in future research, and moreover, researchers could investigate how these IoT-based wearable devices are perceived by people. Similarly, more focus should be on the importance of their design characteristics such as shape, size and also functionalities to determine an effective, optimal, ease device for better usefulness. [47].

## Figures and Tables

**Figure 1:** study and identification of relevant articles flowchart.

**Figure 2:** A look from 1975 to 2021 wearable technologies timeline [18].

**Figure 3:** Feature-based comparison of wearable devices.

**Figure 4:** Different aspects in digital health.

**Figure 5:** A typical intelligent wearable system block diagram.

**Figure 6:** IoT and wearable device architecture.

**Table 1:** Three different stages of AD with their impacts.

SN	AD stages	Things causes by AD
1	Early stage	Having difficulty in speech, memory, work, and social skills or settings. Misplacing or losing a valuable object. Logical and judgmental thinking.
2	Mild stage	Not able to recall some basic information about their phone number, address, and the school they graduated from. Having difficulty in speech, memory, social skills, logical thinking, and senses.
3	Moderate stage	Losing the ability such as dressing themselves where in this stage the patient will be fully dependent on someone such as a caregiver or family member. Require assistance every time, having difficulties in communication, movement, and some other daily activities.

The article "IoT-Based Wearable Devices for Patients Suffering from Alzheimer Disease" was published in 2022. Journal: Contrast Media Mol Imaging.

**Table 2:** Pricing of wearable devices and their availability.

SN	Wearable device	Cost	Availability
1	Smart biomedical system	N/A	N/A
2	Smart glasses	Cost-effective	N/A
3	Smart assistive mhealth system		N/A
4	Environment aware system	N/A	N/A
5	AD-patient monitoring device	40$	N/A
6	Halcyon device	Cost-effective	N/A
7	Intelligent assistive tool	N/A	N/A
8	Autonomous tracking device	Prototype cost ₹750 or $10	N/A
9	Smart assistive glasses	N/A	N/A
10	Smart glasses	N/A	N/A

**Table 3:** Sensors used in wearable devices.

SN	Wearable device	Used sensors
1	Smart biomedical system	Gyroscope, accelerometer
2	Smart glasses	NO
3	Smart assistive mhealth system	NO
4	Environment aware system	3axis accelerometer, HTU21D
5	AD-patient monitoring device	BPM sensor, MPL3115A2 pressure and altitude sensor, ADC, DFRobot heart-rate sensor, bluetooth module
6	Halcyon device	Accelerometer
7	Intelligent assistive tool	Pulse sensor
8	Autonomous tracking device	No
9	Smart assistive glasses	Accelerometer, gyroscope sensor
10	Smart glasses	Microelectromechanical, systems sensor, accelerometers

**Table 4:** Feature comparison of the wearable devices.

SN	Wearable device	Design aspects
1	Smart biomedical system	Implemented and designed with low-cost components but no miniaturize to wearable device
2	Smart glasses	Proposed but not developed the wearable device
3	Smart assistive mhealth system	Implemented and designed components but no miniaturize to wearable device
4	Environment aware system	Wearable waist-bag device
5	AD-patient monitoring device	Not wearable, autodesk FUSION 360 and a 3D printer is used for designing the case and printing it.
6	Halcyon device	Tag is used for detection of patient's engagement with home appliances
7	Intelligent assistive tool	The system built as a prototype
8	Autonomous tracking device	Design approached
9	Smart assistive glasses	Prototype designed
10	Smart glasses	Prototype designed

**Table 5:** Wearable device's location tracking.

SN	Wearable device	Location tracking
1	Smart biomedical system	GPS
2	Smart glasses	No
3	Smart assistive mhealth system	No
4	Environment aware system	GPS
5	AD-patient monitoring device	No
6	Halcyon device	Using the bluetooth tags
7	Intelligent assistive tool	GPS
8	Autonomous tracking device	GPS, geo-fencing
9	Smart assistive glasses	GPS, geo-fencing
10	Smart glasses	BLE gateway

The article "IoT-Based Wearable Devices for Patients Suffering from Alzheimer Disease" was published in 2022. Journal: Contrast Media Mol Imaging.

**Table 6:** Various services provided by wearable devices.

SN	Wearable device	Service 1	Service 2	Service 3	Service 4	Service 5
1	Smart biomedical system	Clock monitoring	Location on the map	Medication time reminder	Emergency call button	Mobile app
2	Smart glasses	Facial perception model is being used in recognizing a person and to extract the features of facial accordingly	Micro database is used for recording the ground truth of facial features of related people around the patient	Matching metric is then used for comparing facial features from a real-time feature		
3	Smart assistive mHealth system	Audiovisual alert	Medication schedule is stored in the nonvolatile memory	e liquid crystal display (LCD) shows the medicine to be taken	Sound effect to get the attention	Sends message to the physician
4	Environment aware system	GPS localization	Environment monitoring	Activity	Fall detection	Mobile app service
5	AD-patient monitoring device	Environmental temperature				
	Atmospheric pressure	Heart pulse	Small screen display	Mobile app service		
6	Halcyon device	Detecting the patient's engagement with home appliances	Instruction assignment	Instruction delivery	Movement tracking	Mobile app service
7	Intelligent assistive tool	Heart rate monitoring	Reminder for taking medicine	Monitoring location of patient's	Finding lost items	Mobile app service
8	Autonomous tracking device	Real-time location tracking	Text message can be sent to the mobile number of caregivers	Alert is sent whenever the patient moves		
9	Smart assistive glasses	Location detection of misplaced objects	Monitoring and guiding the patient for their last seen location	Identification and display of the names of relatives, friends on the AR display	Sending patient location to caregiver simultaneously through SMS	Predicting if patient removed the wearable device and what is the cause
10	Smart glasses	Recognize daily movements				Web-based frontend server used to display

**Table 7:** The user interface of wearable device.

SN	Wearable device	Mobile supported OS	Remarks	Connection
1	Smart biomedical system	Mobile app android	Null	Wi-Fi, Bluetooth, GSM
2	Smart glasses	No	Wearable IoT with complex artificial perception embedding for AD patients	N/A
3	Smart assistive mhealth system	No	For optimal performance, the system can be further miniaturized into a wearable device	GSM, SIM (SMS is used to send message)
4	Environment aware system	Android application	To increase the acceptance, rate the authors stated that the proposed system can be decreased to a smaller size due to the feedback was uncomfortable by many of the patients.	DFRobot GPS/GPRS/GSM shield V3.0
5	AD-patient monitoring device	Software was written into AppInventor	It is suggested by the authors that by using higher performance sensors it can be upgraded, and for reducing the device size a PCB is needed.	Bluetooth
6	Halcyon device	Full-fledged Android 4.2.2 OS is running on the “XTouch-Wave”. Android mobile app	Since there are chances that a patient might takes of the wearable like watch and not wear it again that is where halcyon device can be effective solution	Near field communication (NFC), bluetooth, and RFID (radio frequency identifier‐cation)
7	Intelligent assistive tool	Mobile app	As future work, it is suggested a few more features may be added and developing the system into a wearable device to provide more patient's medical details.	GPS-WiFi
8	Autonomous tracking device	Mobile text on number	In the future, the authors mentioned that more features can be added that are lacked now and improve the system.	GSM
9	Smart assistive glasses	No	The smart glasses were developed as a prototype and suggested to be a practical solution in the future that can help AD patients.	Wi-Fi, bluetooth
10	Smart glasses	Web-based frontend server	Null	BLE (bluetooth low energy) gateway

The article "IoT-Based Wearable Devices for Patients Suffering from Alzheimer Disease" was published in 2022. Journal: Contrast Media Mol Imaging.

**Table 8:** Contrasting between the surveyed wearable devices.

SN	Wearable device	Availability	Cost	Sensor used	IoT	Connection via	Design aspect
1	Smart biomedical system	N/A	N/A	Gyroscope, accelerometer	Yes	GSM, W	Implemented and designed with low-cost components but no miniaturize to wearable device
2	Smart glasses	N/A	N/A	No	Yes	Null	Wearable glasses
3	Smart assistive mhealth system	N/A	N/A	No	No	GSM, SIM	Proposed but not developed the wearable device
4	Environment aware system	N/A	N/A	3axis accelerometerHTU21D	Yes	DFRobot GPS/GPRS/GSM shield V3.0	Wearable waist-bag device
5	AD-patient monitoring device	N/A	40$	BPM sensor, MPL311 A2 pressure and altitude sensor, ADC, DFRobot heart-rate sensor, bluetooth module	Yes	Bluetooth	Not wearable, autodesk FUSION 360 and a 3D printer is used for designing the case and printing it.
6	Halcyon device	N/A	Cost-effective	Accelerometer	Yes	Near field communication (NFC), bluetooth, and RFID (radio frequency Identifi‐cation)	Tag is used for detection of patient's engagement with home appliances
7	Intelligent assistive tool	N/A	N/A	Pulse sensor	Yes	GSM	The system built as a prototype
8	Autonomous tracking device	N/A	Prototype cost ₹750 or $10	No	Yes	GSM	Designed approached
9	Smart assistive glasses	N/A	N/A	Accelerometer, gyroscope sensor	Yes	Wi-Fi, bluetooth	N/A
10	Smart glasses	N/A		Microelectromechanical, systems sensor, accelerometers	Yes	BLE (bluetooth low energy) gateway	Prototype designed

The article "IoT-Based Wearable Devices for Patients Suffering from Alzheimer Disease" was published in 2022. Journal: Contrast Media Mol Imaging.

**Table 9:** Comparison of various wearable devices based on their features.

Product	Design	Features						
		Alert/reminder	Location tracking	Emergency call	Display	Connectivity	Sensor	Mobile app
Smart biomedical system	Wearable embedded	Yes	Yes	Yes	Yes	Wi-Fi, Bluetooth, GSM	Gyroscope, accelerometer	Yes
Smart glasses	Wearable	Yes	No	No	Yes	No	NO	No
Smart assistive mhealth system	System design	Yes	No	Yes	Yes	GSM, SIM card	No	No
Environment aware system	Waist wearable belt	Yes	Yes	Yes	No	Wi-Fi, GSM	3axis accelerometer, HTU21D	Yes
AD-patient monitoring device	Arduino nano-based device	Yes	Yes	No	Yes	Bluetooth	BPM sensor, pressure and environmental temperature sensor	Yes
Halcyon device	Wearable	Yes	Yes	No	No	Wi-Fi, SIM card, GSM, bluetooth	Null	Yes
Intelligent assistive tool	Conceptual design	Yes	Yes	No	Yes	Wi-Fi, GSM	Pulse sensor	Yes
Autonomous tracking device	Wearable embedded	Yes	Yes	No	Yes	GSM	Yes	Yes
Smart assistive glasses	Wearable	Yes	Yes	No	Yes	Wi-Fi, bluetooth	Accelerometer and gyroscope sensor	Yes
Smart glasses	Wearable	Yes	Yes	No	No	BLE (bluetooth low energy) gateway	Microelectromechanical systems sensor, accelerometers	No but display in server

**Table 10:** The basic components of an intelligent wearable device.

Component name	Description
Accelerometer	To keep track of all movements. The velocity and position of an accelerometer sensor are measured inertially [31]. It can detect inclination, tilt, and body orientation on three axes in most cases.
Power battery	Like any other electric devices, wearable devices also require battery power for the device to start functioning. Since wearables are expected to explode in popularity, and many semiconductor vendors are preparing for this by developing new level of battery-management technologies expressly for wearables [32].
Controller	Sensor network nodes and wearable devices are essentially small, attached devices. An analogue signal must be transformed into digital data before it can be broadcast over a wireless network or easily interfaced with other components of the wearable device. This job is done with something called controller or microcontroller that is attached to the wearable, and the main point here is every controller is consumed power so choosing a power efficient controller is the key [33].
Display	Wearable devices include everything from artificial heart monitors to fit bands that can track your daily steps. Many factors have aided this expansion [34], one of those factors is the liquid crystal display (LCD) panels, which enable high resolutions to be achieved even on tiny screens.
Internet	Wearables provide real-time user monitoring, any moment, and anywhere, in the digital-health ecosystem, enhancing care of patient and helping caregivers save time on their administrative works [35]. Wi-Fi plays a major role in wearables if we want to send the data to another system or connect to another platform like Cloud or mobile health application, and so on (The link between the cloud and wearable technology-compare the cloud, n.d).
Cloud computing	Data collection and analysis are at the heart of wearable technology and cloud computing is where one can store this data for further investigations and analysis [36]. Nowadays, cloud computing became an integral part of wearable technology and IoT-based devices [37]
Mobile application	Mobile applications are assistive technologies that are used in monitoring the health of an individual continuously, and these applications can be used in a variety of diseases, including AD (Sarkar and Lacusesta, 2019). There are various mobile health applications that have been developed over the past years for specific diseases like AD to assist and help the patient and their caregivers.

The article "IoT-Based Wearable Devices for Patients Suffering from Alzheimer Disease" was published in 2022. Journal: Contrast Media Mol Imaging.

**Table 11:** List of all the papers with their aims and their future scope and limitations.

Author's name and Ref	Title	Aim	Target stage	Future scope and limitation
(Ahmed and Al-Neami, 2020 [19]) Qayssar a et al.	Smart biomedical assisted system for AD patients	Wearable device and an IoT platform for the caregiver. Provide continual monitoring for AD patient's stability state. Capabilities are a reminder for medication time, location display on the map, emergency button call.	AD patient	—
(Roopaei et al., 2018 [20]) Mehdi et al.	Wearable IoT with complex artificial perception embedding for AD patients	IoT-based wearable glasses. To assist the patient in recognizing and identifying the people in a patient's family, colleagues, friends.	Memory-impaired (early stage)	—
(Temitope O. Takpor, Jimmy ademola, Segun I. Popoola, Joke A. Badejo, 2017) Temitope et al. [21]	Smart assistive system for adherence of medication for AD patients	An intelligent assistive system that can help elderly AD patients in medication adherence by an audiovisual alert and via an LCD to see the right medication at the right time.	Memory loss disability (Mild stage)	For optimal performance, the system can be further miniaturized into a wearable device
(Oliveira et al., 2014)Ana barreto et al. [22]	An environment aware system for AD patients	The aim of the waist-wearable belt device is to monitor the environment humidity and temperature, location and movement of the patient. The caregiver can receive information related to the patient.	Late stage	To increase the acceptance rate, the authors stated that the proposed system can be reduced to a smaller size owing to the feedback from many patients that they were uncomfortable to wear.
(Cazangiu et al., 2018) Teodor cazangiu et al. [23]	Monitoring device for AD patients	A single sensor for environmental temperature, heart pulse, and atmospheric pressure, and generating the output in a screen to display all those health parameters. And those parameters can be displayed in a smartphone using bluetooth.	Moderate stage	In the future, it is suggested by the authors that by using higher-performance sensors, it can be upgraded, and for reducing the device size a PCB is needed.
(Zellefrow et al, 2017) B.Zellefro et al. [24]	Assistive technology for AD patients- (halcyon)	A wearable smartwatch that is bluetooth-based can monitor and track AD patient along with a connected assistive indoor platform, which then can aid the AD patients during the daily routine.	Early stage	—
(Omar et al., 2019) Kazi Shahrukh Omar et al. [25]	An intelligent assistive tool for AD patients	Designed and developed an integrated autonomous system that includes features such as a reminder for taking medicine, heart condition monitoring, constant monitoring of the patients, and finding lost items of patients. For utilization of that feature, a mobile application is also developed.	Moderate stage	The system was built as a prototype and used in an academic environment and therefore, no evaluation study is done with real users. The module of the smart medicine box also has an issue that this cannot work when there is no Wi-Fi connectivity. As future work, it is suggested a few more features may be added and developed in the system of a wearable device to provide more patient's medical details.
(Hegde et al., 2019) Niharika Hegde et al. [26]	An autonomous lower cost tracking device for AD patients	A wearable device using a concept called geofencing and GPS for tracking the real-time location, which can help a caretaker in AD patient tracking has been developed.	Early and moderate stages	In the future, the authors mentioned that more features can be added that are lacking now and improve the system. The intended features to be added are logging of vital signs and monitoring, fall detection, communication in two ways with caregivers. The generated data from these can be used for analyzing and achieving the insights that are useful and can help in providing predictive and preemptive healthcare.
(Gacem et al, 2019) Mohamed ait Gacem et al. [27]	Smart assistive glasses for AD patients	Smart glasses are equipped with an AR screen to perform the basic functions of a caretaker. Features are location and detection of the misplaced object and help out the patient to locate what they have seen last, identifying, and showing the relatives and friends names on the screen, monitoring the patient all the time.	Early and moderate stages	The smart glasses were developed as a prototype and suggested to a practical solution in the future that can help AD patients.
(Chen et al, 2018)Wu-Lin Chen et al. [28]	Smart wearable glasses	Smart glasses is a warning system for behavioral difference for dementia warning and early depression.	Early stage	This wearable device can be useful in recognizing daily movements such as running, walking, standing, lying down, sitting, and many other movements.

The article "IoT-Based Wearable Devices for Patients Suffering from Alzheimer Disease" was published in 2022. Journal: Contrast Media Mol Imaging.

## Data Availability

The data will be available on request.
